This article has been retracted.

# Analysis of Research Status and Development Trend of Nanotoxicology of Liliaceae Medicinal Plants

**DOI:** 10.1155/2022/9777817

**Published:** 2022-07-21

**Authors:** ChaoQun Liu, Yinquan Wang, DongLing Liu, Tao Yang, ZhanWen Tang

**Affiliations:** ^1^College of Pharmacy, Gansu University of Chinese Medicine, Lanzhou 730030, China; ^2^Northwest Collaborative Innovation Center for Traditional Chinese Medicine Co Constructed by Gansu Province & MOE of PRC, Lanzhou 730030, China; ^3^Key Laboratory of Microbial Resources Exploitation and Application Lanzhou, 730000, China; ^4^Institute of Biology Gansu Academy of Sciences, Lanzhou 730000, China

## Abstract

The research status and development trend of nanotoxicology of Liliaceae medicinal plants were analyzed. In the research, the toxicology of Liliaceae medicinal plants was investigated by the preparation method of silver nanoparticles. By means of spectral curve experiment, the present situation of nanotoxicology of Liliaceae medicinal plants was analyzed, and then its subsequent development trend was analyzed. In this process, Liliaceae medicinal plants could be used effectively, which could create great economic benefits. In the application of the above scheme, the toxicological degradation of Liliaceae medicinal plants could be controlled at about 96%. The high-dose silver nanoparticles could reach 100 *μ*M, and the silver nitrate could reach 10 or 30 *μ*M.

## 1. Introduction

Angiosperms are a family of the class monocotyledons. They are usually perennial herbs, but a few are woody or tendril vines. They are bulbous or rhizomes. Leaves are basal or cauline. Cauline leaves are usually alternate and a few opposite or whorled. The leaves of a few species degenerate into scales. Inflorescences are various, usually racemes or cymose umbels or panicles. Flowers are bisexual and radially symmetric. There are 6 petal-like tepals, which are arranged in 2 whorls and separated or united. There are 6 stamens. The ovary is superior and 3-loculed with axial placenta. There are about 240 genera and 4,000 species worldwide. They are mainly in warm regions and tropics. There are 60 genera and 600 species in China, which spread throughout the country. Lily, tulip, hyacinth, day lily, hosta, and asparagus are famous ornamental flowers. The bulb, rhizomes, or whole grass of fritillaria, lily, yellow essence, jade bamboo, anemone, lily of the valley, ophiopogon, and quinoa can be used for medicine. Onions, garlic, cauliflower, leeks, onions, stone pine can be used as condiments. Lily bulbs can be eaten or extracted from starch. Plants often have mucous cells and calcium oxalate needle bundles. There are *x* = 3 − 37 chromosomes. They are herbs with untubed bulb and fleshy scaly leaves. Single leaves are alternate. Flowers are large, with 6 separated tepals and 6 stamens. Anthers are t-shaped. There 3 carpels, which are 3-locular. The stigma is capitate. They are 70~150 cm tall. Stems have purple stripes and are smooth. Leaves are obovate and needle-shaped. The upper leaves are small and 3-5 veined. Flowers are trumpet-shaped, fragrant, and milky white, with slightly purplish on the outside and tips spreading outward or slightly curling. Pollen grains are reddish-brown. Ovary is long terete and stigma is 3 lobed. Capsules are rectangular round and angular. They are born below the altitude of 900 m on the hillside grass, stone crevices, or near the cottage. They are distributed in Hebei, Henan, Shanxi, Shaanxi, Anhui, Zhejiang, Jiangxi, Hubei, Hunan, and other places (see Figure 1).

## 2. Literature Review

Pyrrolizidine alkaloid is the most important toxic natural product after aristolochic acid [1]. There are more than 350 PAs in more than 6,000 plant species, accounting for 3% of the world's total flowering plants. The symptoms of the acute toxicity caused by PAs is mainly hemorrhagic liver necrosis, giant hepatocellular disease caused by low dose and long-term inhalation, hepatic pulmonary vein obstruction, biliary epithelial cell proliferation, and cirrhosis. Among people with acute PAs poisoning, about 20% will die. About 50% recover fully within a few weeks. And about 20% progress to chronic venous obstruction and cirrhosis with a process that takes years. Others develop into subacute venous obstruction. According to the epidemiological investigation, in South Africa, Afghanistan, Jamaica, India, the former Soviet Union, and other countries, a large number of liver diseases are related to the consumption of cereals, beverages, and herbs containing PAs [2]. The planting area of lily in each region is shown in Figure 2.

With the rapid development of nanotechnology and the increase of nanomaterials, the safety of nanotechnology is attracting worldwide attention. Nanomaterials can enter the natural environment through a variety of ways and produce a variety of environmental behaviors, which may cause toxic effects on the organism. And its ecological impact cannot be ignored. At present, the international research on the ecological effects of nanomaterials, especially the environmental behavior, is still in its infancy. There are very few valuable research results, and there are still many uncertain ecological security issues to be further investigated. Based on the summary of relevant research at home and abroad, the source of nanomaterials, the way of entering the environment, environmental behavior, ecotoxicological research status, and the contents to be further investigated were briefly reviewed [3]. The development process of nanotechnology is shown in Figure 3.

Nowadays, nanotechnology is developing rapidly all over the world. Nanomaterials have a wide range of applications in electronics, magnetism, optics, biomedicine, pharmacy, cosmetics, energy, sensors, catalysis, and materials science. It is predicted that the global market value of nanotechnology related products will reach $1 trillion by 2015, with 2 million workers. With the development of more and more new nanomaterials and the marketing of nanoproducts, the contact objects and contact opportunities of nanomaterials or nanoproducts increase greatly. And the safety of nanotechnology has attracted worldwide attention. Some nanomaterials such as single-walled carbon nanotubes can achieve a variety of tissues of animals, such as the heart, liver, spleen, lung, kidney, stomach, brain, bone, muscle, small intestine, skin, and blood. Fe_2_O_3_-Glu nanoparticles can even reach the eyes and gonad tissue. Nanomaterials can penetrate the blood-brain barrier, blood eye barriers, and blood testosterone barrier, which may endanger the safety of the organism. Existing researches have shown that nanomaterials can affect organisms at the cellular level, subcellular level, gene level, protein level, and overall animal level. As the basis of life activity, the importance of ecological environment is obvious. Whether and to what extent nanomaterials will affect the ecological environment is a very important part of the safety of nanotechnology [4]. The application fields of nanotechnology are shown in Figure 4.

## 3. Research Methods

There are many factors affecting the biological toxicity of silver nanomaterials, including their physical and chemical properties and environmental conditions. Size has an important influence on the interaction mode of silver nanomaterials with body cells, the uptake rate of silver nanomaterials by cells, and the cytotoxicity of cells [5]. When the size of silver nanoparticles is large, they enter cells mainly through phagocytosis and macropinocytosis. Otherwise, it is mainly through endocytosis. Second, small silver nanoparticles are more likely to enter cells and accumulate than large ones. In addition, Chen et al. found that silver nanoparticles with a particle size of 15 nm were more cytotoxic than silver nanoparticles with a particle size of 50 and 100 nm. Shape also plays a key role in the biotoxicity of silver nanomaterials. Researches have shown that spherical silver nanomaterials get into cells more easily than other shapes. Compared with spherical silver nanoparticles and silver nanowire, silver nanocubes are less toxic to model plants. Surface charge has a certain influence on the reaction between silver nanomaterials, ions, and biomolecules. And it also determines the colloidal behavior of silver nanoparticles. By influencing the aggregation behavior of silver nanoparticles, the toxic response of cells to them is changed [6]. Researches have shown that the positively charged silver nanoparticles toxicity is more toxic than the negatively charged ones. It is because the positively charged silver nanoparticles combine with the negatively charged cell membrane phospholipids head or protein structure more easily, which causes the mechanical damage of the cell membrane, leading to more silver nanoparticles into the cells and even cell death. Surface charge also has a certain influence on the biological distribution of silver nanoparticles. For example, Long et al. found that negatively charged silver nanoparticles could cause the lysis of plasmic prokinin releasing enzyme in mice, thus affecting its distribution in mice, while neutral or positively charged silver nanoparticles have no effect [7]. The dose response curve of silver nanoparticles is shown in Figure 5. The dose response of single strain to silver nanoparticles is described in Table 1.

The biological distribution of silver nanoparticles is also closely related to their exposure dose. A large number of researches have shown that the distribution and accumulation of silver nanoparticles in organism are dose-dependent. The higher the dose is, the more negative the effect is. But sublethal exposure doses of silver nanoparticles greatly promote the growth of microorganisms, showing a certain stimulation effect. It also suggests that the poison excited response of the microbes to the silver nanoparticles [8]. The exposure dose of silver nanoparticles also has a very important effect on their toxicity. Although the toxicity of silver nanomaterials and Ag + is dose-dependent, their uptake pathway and intracellular behavior are different. Compared with Ag+, silver nanoparticles have a stronger ability to penetrate biological barriers [9]. Some researchers found that when rats were exposed to silver nanoparticles, their distribution in the blood, kidneys, liver, lungs, olfactory bulb, and brain was dose-dependent. After 28 d of continuous administration, it was found that cholesterol value and alkaline phosphatase of rats showed a significant dose-dependent trend. And silver nanoparticles higher than 300 mg·kg^−1^ led to slight liver injury [10]. However, more researches have reported the dose response of single bacteria to silver nanoparticles. The preparation of silver nanoparticles is shown in Figure 6.

pH can affect the dissolution and stability of silver nanoparticles. *pH* = 6. And the electrophoretic mobility of silver nanoparticles is shown in Formula (1):

(1) $$\begin{array}{c} ca=2{cm}^{2}\cdot v^{-1}\cdot s^{-1}. \end{array}$$

When *pH* = 7.5\9, its electrophoretic mobility is as shown in Formula (2):

(2) $$\begin{array}{c} ca-3.5{cm}^{2}\cdot v^{-1}\cdot s^{-1}. \end{array}$$

In the presence of acidic substances, pH also affects the surface charge of silver nanoparticles. Adegboyega et al. studied the effect of pH on the toxicity of silver nanoparticles. The results showed that silver nanoparticles had high toxicity to Pseudomonas fluorescens at low pH. However, an increase in pH results in a decrease in the cytotoxicity of silver nanoparticles. Environmental ligands can react with Ag + to form relatively stable substances, which not only affects the bioavailability of Ag+, but also affects the toxicity of silver nanoparticles to a certain extent. Inorganic ligands such as Cl- can be used as scavenger to increase bacterial activity [11]. The Ag + release capacity of silver nanoparticles is also affected by environmental ligands.

### 3.1. Preparation of Silver Nanoparticles

In the research, silver nanoparticles needed in the experiment were synthesized by referring to the method of Deokar et al. and sodium citrate was used as stabilizer [12]. 0.6 mM sodium citrate and 1.8 mM sodium borohydride were dissolved into 59.5 mL ultrapure water, which was stirred vigorously under ice bath condition. Then, 0.5 ml 24mMAgNO_3_ solution was quickly added to the above mixed solution and stirred evenly. At this time, the mixed solution turned yellow, indicating the formation of silver nanoparticles. After 3 min, the ice bath environment was removed, and the stirring was continued at room temperature for 3 h [13]. The synthesized silver nanoparticles were needed to be purified using 1 KDa regenerated cellulose membrane to remove excess chemical components, such as sodium citrate and Ag+, for reserve. After filtration by ultrafiltration centrifuge tube, the concentration of Ag + in the filtrate was measured by ICP-OES to determine the dissolution degree of silver nanoparticles (the dissolved part of silver nanoparticles solution in suspension was less than 1%) [14]. The concentration of silver nanoparticles was needed to be digested by nitric acid and hydrogen peroxide solution and then determined by flame atomic absorption spectrometer. The specific research ideas of the research are shown in Figure 7.

After the silver nanoparticles were uniformly dispersed by ultrasonic dispersion method, the solution of 3−3.5 mL silver nanoparticles was placed in a quartz colorimetric plate. And the plasma resonance absorption peak was measured by UV-Vis spectrophotometer in the wavelength range of 200−700 nm to determine whether the silver nanoparticles coated with sodium citrate were successfully synthesized [15]. The hydrodynamic diameter and zeta potential of silver nanoparticles could be determined by the dynamic light scattering (Zetasizer Nanoseries Nano-ZS90, Malvern Instruments, UK). The size, morphology, and particle distribution of silver nanoparticles could be analyzed by JEOLJEM-3010 transmission electron microscope. Firstly, the silver nanoparticle solution was ultrasonic dispersed for 3 min, and then the sample solution was dropped onto the microsol for natural air drying under indoor conditions. Subsequently, electron microscope images were taken under 200 kV acceleration voltage and the size of silver nanoparticles could be analyzed by software “NanoMeasurer1.2.5” [16].

White rot fungi were used in the experiment. Phanerochaete chrysosporium BKMF-1767 was purchased from Chinese Typical Culture Storage Center. Kirk medium was used for the cultivation of chrysosporium in the research. And the formula (L-1) is as follows: 0.01 g CaCl_2_, 0.05 g MgSO_4_·7H_2_O, 0.2 g kh_2_PO_4_, 0.221 g ammonium tartrate, 1.641 g anhydrous sodium acetate, 11.098 g glucose, 0.5 mL vitamin solution, and l mL inorganic solution [17]. Specifically, spore suspension with a concentration of 2 × 106/mL was added to 200 mL of the above medium and then placed in a constant temperature oscillation incubator to cultivate at 37 °C and 150 rpm to form mycelium pellets [18].

After incubation for 72 h, phanerochaete chrysosporium was centrifuged for 5 min at a rate of 10,000 × *g*. Also, remove the top layer to remove the mycelium and then wash several times with NaHCO3 buffer solution (2 mM). This negative effect has no effect on the bioavailability of the silver and has been chosen as the median accuracy because it can bind to AgNPs/Ag + and avoid precipitation ligands and other interferences [19]. In addition, dilute the storage of silver nanoparticles with 2 mM Na2HCO3 solution to obtain the concentration of silver nanoparticles required for the test (0 *μ*M, 1 *μ*M, 10 *μ*M, 30 *μ*M, 60 *μ*M, and 100 *μ*M), when time initial concentration was 2,4-DCP stored at 20 mg/l in solution. Add the same amount of micelles (0.6 g/l) to the solution, and incubate at 37 °C in an incubator at 150 rpm. The response to AgNO3 was similar [20].

To determine the effect of 2,4-DCP concentration on the absorption and degradation activity of P. flavorosa, 0.6 g/l mycelium of P. flavorosa was cultured at different levels respectively. At this time, the initial concentration of AgNP in solution was 10 *μ*M. The concentration of 2,4-DCP in solution can be determined by liquid chromatography (HPLC, Agilent1100), and the biodegradable intermediates of 2,4-DCP can be determined by GCMS-QP2010Ultra equipments, with RTX-5 capillary column [21].

The pH in the solution was measured by pH meter and the experimental data were recorded. The extracellular protein content of phanerochaete chrysosporium was determined by Coomassie Brilliant Blue method. The sample solution was first taken into a centrifuge tube and then centrifuged. And 1 mL supernatant was taken into 5 mL Coomachus Bright Blue G250 solution, mixed evenly, and stood for 3 min at room temperature. Then, the extracellular protein content was analyzed by UV spectrophotometer at 595 nm [22].

### 3.2. Discussion of Results

The morphology and size of silver nanoparticles are determined by a conductive electron microscope. The AgNPs prepared were monodispersed spherical particles with an average particle size of 11.9 ± 9.4 nm. AgNPs had a strong characteristic absorption peak of plasma resonance at the wavelength of 395 nm, and the zeta potential of AgNPs in ultrapure water was −30.9 ± 2.3 mV. In addition, according to the analysis of dynamic light scatterometer, the hydrodynamic particle size of AgNPs was 20.2 ± 0.3 nm. By comparing the particle size measured by transmission electron microscope and dynamic light scatterometer, it could be seen that there was a large difference between them, which may be caused by different sample preparation processes [23]. TEM images depicted the nuclear particle size of the sample in the dry state, while the particle size measured by dynamic light scatterometer included the nuclear particle size of the particle and its expanded surface corona particle size. So the hydrodynamic particle size of AgNPs was slightly larger than that measured by TEM. The plasma resonance absorption spectrum is shown in Figure 8.

When Phanerochaete chrysosporium was exposed to AgNP ions, the degradation activity of 2,4-DCP was reduced depending on the dose. When the initial concentration of AgNP was between 0 and 60 *μ*M, treatment with AgNPs had little effect on the degradation of 2,4-DCP and maintained a high degradation rate (>96%). However, when the AgNP concentration was increased to 100 *μ*M, the degradation rate of 2,4-DCP decreased to 73.38%. In addition, phanerochaete chrysosporium was found to reach 100% degradation level of 2,4-DCP when exposed to only 2,4-DCP (without AgNPs) [24]. This suggests that low doses of 2,4-DCP (20 mg/l) do not affect the bioactivity of phanerochaete chrysosporium, which is according to our previous report. Changes in total silver content indicate that AgNP and other materials have moved from the fluid phase to the biophase and that organic acids and intracellular proteins are involved in biological processes involved. Affect the exchange rate of the total amount. When Phanerochaete chrysosporium is exposed to low concentrations of AgNP, the removal rate of total silver was significantly increased (96.11%, 99.63%, and 94.17% when the initial AgNPs concentrations were 10 *μ*M, 30 *μ*M, and 60 *μ*M, respectively). However, when the AgNPs concentration was 1 *μ*M, no silver content could be detected after 12 h. In contrast, when 100 *μ*M AgNPs was used to treat phanerochaete chrysosporium, the removal rate of total silver was only 37.35%.

High concentrations (100 *μ*M) of AgNP reduced the release of both 2,4-DCP and total, leading to disease, apoptosis, and cell death due to high cytotoxicity AgNP. Studies have shown that the toxic processes of AgNPs include AgNPs themselves or AgNP releases, which include membrane integrity, slow cell cycle, ROS production, energy metabolism. Thus, the degradation of 2,4-DCP and the absorption and distribution of AgNP and Ag + were affected by AgNP toxicity [25].

In addition, as the concentration of AgNP increased in the range of 1 *μ*m-60 *μ*M, the total absorption capacity increased linearly from 0.02 mg/g to 1.00 mg/g. However, when the AgNPs are at their maximum, the total absorption begins to decline. The increase in total adsorption capacity is due to the high concentration of AgNP, which may be due to the effectiveness of overcoming the major changes in phanerochaete chrysosporium and liquid phase and thus the presence of most of the collisions of phanerochaete chrysosporium. AgNPs and Ag + also have a higher penetration rate to better absorb total reserves. Excess AgNPs are saturated at some binding site, which reduces cell absorption. However, as the concentration of AgNP increases, the degradation capacity of 2,4-DCP first reaches equilibrium and then decreases. This may be due to the fact that high levels of AgNP inhibit the decomposition of chrysosporium phanerochaete.

In conclusion, data suggest that AgNP-induced cytotoxicity is the dose. For example, high doses of AgNPs (100 *μ*M) increased cytotoxic effect. In addition, low concentrations of AgNP were recommended to improve microbial bioactivity and adaptability, facilitating the simultaneous elimination of 2,4-DCP and total bonds. However, when exposed to high concentrations of AgNP, the efficiency of 2,4-DCP removal and total yield was reduced. The activating effect of AgNPs 2,4-DCP, and total excretion may be due to the fact that low doses of AgNP (e.g., 1-60 *μM*) phanerochaete activate the toxic healing mechanism of chrysosporium and lead to overcompensation of AgNP.

## 4. Experiment Methods for Verifying the Scheme

It is well known that the release of Ag + plays an important role in the transformation of AgNPs in the aqueous environment and the oxidation process of nanoparticles in solution requires exposure to air and acidic conditions, as shown in Formulas (3) and (4):

(3) $$\begin{array}{c} 4{AG}^{0}+o_{2}⟶2{AG}_{2}o, \end{array}$$

(4) $$\begin{array}{c} 2AG_{2}o+4H⟶4AG^{+}+2H_{2}o. \end{array}$$

The differences and variability of Ag + release patterns in the presence of phanerochaete chrysosporium were investigated. It was found that the metabolic state of phanerochaete chrysosporium could affect the concentration of dissolved oxygen, the pH value of solution, and the production of secretions. It also could remove the surface coating materials of AgNPs and enhance the dissolution gradient of AgNPs by combining with the released Ag+. DO was sufficient in biological systems and was provided by culture at 150 rpm. In addition, enhanced dissolution of AgNPs had been reported at lower pH. In the research, lower pH did contribute to Ag + release to a certain extent. On the contrary, when pH value increased, the release of Ag + in the corresponding water system decreased at lower 2,4-DCP concentration. The release amounts of nanoparticles with different concentrations are shown in Figure 9.

When the initial concentration of AgNP is low, AgNP is slightly heavier; thus, the soluble surface area increases, which in turn increases the rate of Ag + release. When initial AgNPs are low, liquid Ag + concentrations are sometimes high, but Ag + emissions are generally low. Natural organic matter (NOM) has been reported to increase the bioavailability of nanoparticles, improve repulsion of nanoparticles, and thus inhibit Ag + release by AgNP. In addition, special proteins released by P. chrysosporium have the same effect of AgNP as NOM. It may also interact with organic acids formed during metabolism and degradation of 2,4-DCP. Some organic acids act as a source of AgNP, blocking the junctions possible and blocking the continuous flow of AgNP. In this case, the soluble Ag + in the body may be absorbed by the fungal mycelium and interact with the intracellular protein. In these cases, Ag + has been shown to bind to silver-sulfur nanoparticles, thus detoxifying Ag +. In addition to the formation of silver complexes, the reduction in Ag + emission concentrations may be related to the reduction of the reaction of the hydroxyl group in the polysaccharide and the synthesis of the original AgNP. The changes of extracellular protein content under different concentrations of silver nanoparticles are shown in Table 2.

Numerous studies on the toxicity of AgNP have shown that the release of Ag + has a significant effect on the drug toxicity of AgNP. However, studies have shown that the solubility of AgNPs is lower than that of most other solutions, suggesting that the toxicity of AgNPs to chrysosporium phanerochaete may be due to the specific effect of AgNP. Another explanation is that small amounts of AgNP can enter cells and enter the cellular system by endocytosis or macropinocytosis. The tiny cell size releases high levels of metal ions that can disrupt cell function, indicating that a “Trojan horse” interferes with AgNP. The difference in change in Ag + solution was the same starting at 2,4-DCP concentrations as when treated with AgNPs. Under these circumstances, except for 0 mg/l and 80 mg/L2, no significant change in Ag + concentration was observed in 4-DCP, which may be due to the absence of organic matter. Acids obtained from 2,4-DCP to prevent cracking. On the other hand, higher concentrations of 2,4-DCP will affect enzyme activity to change the availability of Ag +.

Figure 10 shows the toxicity of Ag + at different AgNO_3_ concentrations. Ag + showed different cytotoxicity at lower and higher AgNO_3_ concentrations as follows. After exposure to 0.01 *μ*M, 0.1 *μ*M, 1 *μ*M, and 10 *μ*M AgNO_3_ 60 h, the degradation rate of 2,4-DCP was up to 100%. However, the degradation rate of 2,4-DCP after exposure to 30 *μ*M AgNO_3_ 12 h was 22.62%. Under the condition of low AgNO_3_ concentration, the removal rate of total silver was higher than 90%, while under the condition of high AgNO_3_ concentration, the removal rate of total silver decreased. Here, the underlying mechanism of Ag + toxicity may be ROS production and the inactivation of sulfhydryl proteins. In addition, under high concentration AgNO_3_ exposure, the removal rate of total silver decreased with the increase of time. It was speculated that this might be because the exposure of Ag + led to the apoptosis of fungal corpuscular cells, causing part of Ag + to infiltrate from the corpuscular cells. In general, the toxicity of AgNO_3_ was positively correlated with Ag + concentration and the exposure time. The changes of extracellular protein content under different concentrations of silver nitrate are shown in Table 3.

Compared with AgNPs with the same concentration of silver, AgNO_3_ was generally more toxic in biological systems, which may be due to the high uptake potential and bioavailability of AgNO_3_, as well as its complete dissociation, leading to the rapid release of a large amount of free Ag+, while AgNPs slowly released a lower level of ionic silver. The negatively charged fungal cell walls bound to Ag + more easily than negatively charged AgNPs. Ag + had a high affinity for sulfur-containing proteins in the cell membrane and cytoplasm and could bind to phosphoric acid containing molecules such as DNA to damage cells. However, free transport of Ag + across cell membranes and biological barriers was relatively difficult. As for AgNPs, previous researches showed that nanoparticles had stronger transfer ability in cells and even in the nucleus, which could directly interact with key components in cells. It had a strong inhibition effect on RNA transcription through direct binding with RNA polymerase, showing the particle-specific toxicity of AgNPs to a certain extent.

### 4.1. Results

Studies have shown that low concentrations of AgNP affect the degradation of 2,4-DCP in the presence of chrysosporium phanerochaete, and the degradation efficiency of 2,4-DCP (>96%) received. Under acidic conditions, the efficiency of total removal is high. In contrast, phanerochaete chrysosporium is more susceptible to high concentrations of AgNP (100 *μ*M) and also lower concentrations of AgNO3 (10 *μ*M and 30 *μ*M) because it significantly inhibited degradation and excretion of 2,4-DCP. In addition, in this study, the effect of AgNP on Trojan horse could be due to nuclear effect, ionic effect, or both. However, more research is needed to determine which is more effective. One possible cause for the achievement of 2,4-DCP is chlorination and reaction with hydroxyl radicals. The conversion and depletion of Ag + to Ag0 are associated with groups containing amines, carboxyls, carbonyls, and sulfur. The results of these experiments will help to better understand the toxicity of AgNPs and how AgNPs control the breakdown of chlorophenol.

Under 2,4-DCP and AgNPs stress, the accumulation of oxalic acid increased, accompanied by higher MnP and LiP activities. EPS and extracellular proteins were also elevated in response to toxic-induced oxidative stress. However, Ag + introduced with AgNPs to some extent inhibited the production of all tested extracellular secretions compared with AgNPs alone. In addition to the response analysis of extracellular secretions to Ag + and AgNPs combined stress, SEM, HAADF-STEM ,and EDX data also indicated that the toxicity of AgNPs to P. flavoropsis was caused by the added nanoparticles themselves, rather than the AgNPs biosynthesized by Ag + reduction. It was also found that the introduction of Ag + enhanced the particle-specific cytotoxicity of AgNPs in a concentration-dependent manner.

## 5. Conclusions

In the whole exposure process, SOD activity induced by AgNPs was higher. And the catalytic activity of SOD led to the accumulation of H_2_O_2_, thus inhibiting the activity of CAT. When Phanerochaete chrysosporium was exposed to low concentrations of 2, 4 − *DCp*(153*μM*) (7), *AGPS*(≤30*μM*) (8), *AG*^+^(≤*μM*)48 − 72*h* (9), and 11.9 ± 9.4*nm* (10), CAT activity was higher to a certain extent than that at 2−24 h. However, higher concentrations of toxic substances significantly inhibited CAT activity. These experiment results were consistent with observations. Researches showed that the recovery time of cell growth and proliferation under low dose stress was shorter than that under high dose stress. Cellular recovery implied an effective adaptive response of the microbe to a toxic substance, which indicated the production of more enzymes to repair oxidative damage. Compared with the control group, it took a longer time to recover the enzyme activity if the enzyme activity was still inhibited under stress conditions or the enzyme activity could not be repaired under high dose and long-term exposure conditions.

## Figures and Tables

**Figure 1:** Nanotoxicology of Liliaceae medicinal plants.

**Figure 2:** Planting area of lily.

**Figure 3:** The development process of nanotechnology.

**Figure 4:** Application fields of nanotechnology.

**Figure 5:** Dose response curve of silver nanoparticles.

**Figure 6:** Preparation of silver nanoparticles.

**Figure 7:** Research ideas.

**Figure 8:** Plasma resonance absorption spectrum.

**Figure 9:** Nanoparticle release amounts at different concentrations.

**Figure 10:** Comparison of nitric acid concentration.

**Table 1:** Dose response of single bacteria to silver nanoparticles.

Strain	Dose (mg/L)	Lower cell density
Staphylococcus aureus	0.03	Lower cell density
Escherichia coli	−3.6 × 10^−3^	At higher dose
Nitrosomonas europaea	0.002−2	Growth over 100% at certain doses, depending on pH and presence of humic acids
Pseudomonas stutzeri	0.0025−5	Ammonia monooxygenase gene sup regulated when 0.0025 mg/L was used
Azotobacter vinelandii	4	Strain dependent minimum inhibitory concentration (MIC)
Arthrobacter globiformis	12	Inhibition ratio increase with dose; inhibition-dose curve flattens at higher dose
Azotobacter vinelandii	0.1−100	Slower growth rate at higher concentration

**Table 2:** Changes of extracellular protein content under different concentrations of silver nanoparticles.

AgNPs concentrations (*μ*M)	1 h	12 h	24 h	36 h
0	71.67	67.63	66.28	65.79
1	73.92	66.63	66.61	64.09
10	71.67	71.87	75.36	71.57
30	73.09	78.58	79.42	64.36

**Table 3:** Changes of extracellular protein content under different concentrations of silver nitrate.

AgNO_3_ concentrations (*μ*M)	1 h	12 h	24 h	36 h
0.01	71.03	65.68	66.27	64.29
0.1	72.50	59.65	65.36	64.42
1	71.60	65.61	64.91	63.74
10	70.78	66.82	68.28	68.10

## Data Availability

The labeled data set used to support the findings of this study is available from the corresponding author upon request.
